The article "pH Responsive Polymer Micelles Enhances Inhibitory Efficacy on Metastasis of Murine Breast Cancer Cells" was retracted in 2023. Reasons: duplicated images; signs of a paper mill; original data or images not available; unreliable results or conclusions.

# pH Responsive Polymer Micelles Enhances Inhibitory Efficacy on Metastasis of Murine Breast Cancer Cells

**DOI:** 10.3389/fphar.2018.00543

**Published:** 2018-05-23

**Authors:** Jie Wang, Gejing De, Qiaoxin Yue, Hai Ma, Jintang Cheng, Guangwei Zhu, Maobo Du, Hong Yi, Qinghe Zhao, Yanjun Chen

**Affiliations:** Institute of Chinese Materia Medica, China Academy of Chinese Medical Sciences, Bejing, China

**Keywords:** micelles, 4T1, tumor metastasis, paclitaxel, poly(β-amino ester)

## Abstract

A pH sensitive micellar cargo was fabricated for pH triggered delivery of hydrophobic drug paclitaxel with pH controlled drug release profiles. The size, drug loading content, and encapsulation efficiency of PTX loaded micelles were 20–30 nm, 7.5%, 82.5%, respectively. PTX loaded PELA-PBAE micelles could enhance the intracellular uptake of a model drug significantly, with increased cytotoxicity and inhibition of tumor metastasis on 4T1 cells, as confirmed by wound healing assay and tumor cells invasion assay. The expression of metastasis and apoptosis correlated proteins on 4T1 cells decreased remarkably after intervention by PTX loaded polymer micelles, as demonstrated by western blotting and quantitative reverse transcriptional-polymerase chain reaction (qRT-PCR). Our results demonstrated the pH responsive polymer micelles might have the potential to be used in the treatment of metastatic breast tumors.

## Introduction

Tumor metastasis is a major challenge in the treatment of cancer, which accounts for over 90% of mortality of cancer patients due to its metastatic nature and the resistance of the disseminated cancer cells to the current anti-cancer drugs (Valastyan and Weinberg, 2011; Clarke et al., 2015). Among that, breast carcinoma is a major cause of cancer mortality in women as a result of metastasis to other organs (Weigelt et al., 2005). In 2016, breast cancer among women accounts for about 25% of all cancer types and 15% of all cancer mortality was reported in the United States (Siegel et al., 2016). In many cases, metastatic cancers are still incurable using current therapeutic technologies. The progression of cancer metastasis includes the invasion of tumor cells into the surrounding tissues, migration or penetration of the cells through the walls of circulation system, transportation of cancer cells through circulatory and/or lymphatic system, hosting of the metastatic cells at secondary tissues, and extravasation at secondary sites for proliferation (Chambers et al., 2002; Fidler, 2003).

Taxanes are among the most efficacious chemotherapy agents against metastatic breast cancer (Ghersi et al., 2015). Paclitaxel (PTX), as a member of taxanes, is commonly used for the treatment of breast tumor, lung cancer and ovarian carcinoma, etc. (Nehate et al., 2014). However, including PTX, one of the major drawbacks of the current chemotherapeutic strategy is the strong collateral damage to healthy tissues due to the lack of specificity and sensitivity of drug delivery system. Over the past three decades numerous research works had been conducted for the development of cremophor free PTX formulations to eliminate the undesired side effect (Nehate et al., 2014). Various PTX formulations employing nanoparticles (Min et al., 2015), liposomes (Dyondi et al., 2015), micelles (Kim et al., 2004), polymer-drug conjugate (Yang et al., 2014), dendrimer (Khandare et al., 2006), as well as carbon nanotubes (Tavakolifard et al., 2016) as nanocarriers with alleviated systemic toxicity were reported to achieve active or negative targeted delivery of PTX to tumor sites. Among the different anti-cancer drug carriers, polymeric micelles have received considerable attention for developing optimized drug delivery systems during the past decade due to their superior properties such as biocompatibility, biodegradability, elongated circulation time, and tumor accumulation (Suarato et al., 2016; Yan and Li, 2016).

In this article, we employed a pH sensitive poly(β-amino ester) copolymer micelles to entrap PTX for improved inhibitory effect on the metastasis of a murine breast cancer cells. The drug loaded micelles could release their cargo in an accelerated manner under mimic tumor microenvironment conditions. The pH sensitive PTX formulation could effectively inhibit the migration and invasion of tumor cells and increase the sensitivity of PTX on 4T1 cells, as compared with the commercial available drug formulation. The pH responsive polymer micelles are envisaged to have the potential for enhanced chemotherapeutic treatment and reduced deleterious side effects.

## Materials and Methods

### Materials and Cell Lines

Methoxy poly(ethylene glycol) (MPEG, Mw2000), tin (II) 2-ethylhexanoate, and Hoechst 33342 were provided by Sigma-Aldrich (St. Louis, MO, United States). 1,6-Butanediol diacrylate and coumarin-6 (C_6_) were purchased from TCI (Tokyo, Japan). D,L-lactide was produced by Ji’nan Daigang (Ji’nan, Shandong, China). Paclitaxel (PTX) and 1-amino-4-methylpiperazine (AMP) were provided by Adamas (Shanghai, China). PTX injection is a PTX commercial product obtained from Aosaikang Pharm. Co (Nanjing, Jiangsu, China). 3-(4,5-dimethylthiazol-2-yl)-2,5-diphenyltetrazolium bromide (MTT), fetal bovine serum (FBS), trypsin-EDTA and RPMI-1640 medium (RPMI) were obtained from Sijiqing Biotech Company (Hangzhou, China). All other chemicals were of analytical grade and were used as received. Mouse 4T1 breast cancer cells (the Cell Resource Center of the Institute of Basic Medical Sciences, Chinese Academy of Medical Sciences, Beijing, China) were used and maintained in RPMI-1640 medium supplemented with 10% fetal bovine serum (FBS) and 1% penicillin–streptomycin at the circumstance of 37°C, 5% CO_2_ and 95% humidity.

### Polymer Synthesis

Amphiphilic block copolymer poly(ethylene glycol)-*b*-poly(lactide) (PELA) was prepared through ring opening polymerization of D,L-lactide as initiated by MPEG (Heald et al., 2002). Poly(ethylene glycol)-*b*-poly(D,L-lactide)-*b*-poly(β-amino ester) (PELA-PBAE) was acrylated by activation of PELA with acryloyl chloride with following Michael addition of diacrylate ester and piperazine derivates (Chen et al., 2017). Briefly, 6.94 mmol of D,L-lactide was dissolved in 5 mL anhydrous toluene and was polymerized with 0.5 mmol of MPEG as initiator and Tin (II) octoate as catalyst at 130°C for 24 h. The copolymer PELA was obtained by precipitation in diethyl ether and vacuum drying (yield 92%). Next, 0.5 mmol of PELA was dissolved in 5 mL dichloromethane (DCM) and was activated by dropwise adding of 0.6 mmol of acryloyl chloride at 4°C and reacted overnight. The terminal activated PELA was purified by dissolution/precipitation for 3 times by DCM/diethyl ether and vacuum dried (93%). For PELA-PBAE synthesis, 0.5 mmol of acrylic ester terminated PELA was dissolved in toluene and was reacted with 5 mmol of diacrylate and 5.5 mmol of AMP at 50°C for 24 h. The final product PELA-PBAE was obtained by precipitation/dissolution in diethyl ether/DCM thrice and vacuum drying (yield 89%).

### Fabrication of PTX Loaded Micelles

The PELA or pH-responsive PELA-PBAE polymer micelles were prepared by the thin-film hydration according to previous protocol (Chen et al., 2017). In short, PELA or PELA-PBAE and PTX were mixed with predetermined weight ratio and were dissolved in acetonitrile. Then the solvent was evaporated using a RE2000 rotary evaporator (Yarong, Shanghai, China) in a round-bottomed flask at 50°C for 1 h to allow the formation of a thin solid film. The film was then hydrated by de-ionized (DI) water under vigorous shaking on a mini-shaker. The solution was filtrated through Millipore 0.22 μm filter and was lyophilized. Coumarin-6 (C_6_) loaded PELA or PELA-PBAE micelles were prepared according to similar protocols as mentioned above. The size and zeta potential of the formed micelles were measured on a Malvern Zetasizer Nano ZS90 (Worcestershire, United Kingdom) with a detection angle at 90°. The drug loading content (LC) and encapsulation efficiency (EE) were determined by high performance liquid chromatography (HPLC, Shimadzu LC-20A, Kyoto, Japan) equipped with a TOSOH C_18_ column (4.6 × 250 mm, 5 μm, column temperature 30°C), with a triple mobile phase of methanol/acetonitrile/water (35:40:25) and a flow rate of 1.0 mL/min. A fixed amount of lyophilized micelles was dissolved in methanol and subjected to HPLC detection via a UV detector at 227 nm, as compared to a calibration curve of PTX in the mobile phase. The LC and EE were calculated according to the following equations:


$$LC=\frac{\text{weight of drug in the micelles}}{\text{weight of drug loaded micelles}}\times 100\%$$

$$EE=\frac{\text{weight of drug in the micelles}}{\text{weight of the added drug}}\times 100\%$$

### *In Vitro* Drug Release

The release of PTX from micelles was performed according to a protocol reported previously (Chen et al., 2017). In short, 1 mL of PTX-loaded micelle solution was sealed in a dialysis bag (MWCO 3,500) and incubated in 15 mL of phosphate buffered saline (PBS) at pH 7.4 or pH 6.5. The drug release was carried out at 37°C in an incubator shaking horizontally at 100 rpm. The release medium was completely removed and supplemented with fresh PBS at predetermined time intervals. The PTX concentration in the medium was recorded with HPLC with a UV detector operated at 227 nm. The cumulative drug release was integrated from each measurement.

### *In Vitro* Cellular Uptake

Confocal laser scanning microscopy (CLSM) and flow cytometry analysis were carried out to monitor the intracellular uptake and distribution of micelles. For CLSM observation, 1 × 10^5^ 4T1 cells in 500 μL RPMI 1640 were seeded onto glass coverslips which were placed in 12-well plates and incubated for 24 h. Then the cells were incubated with C_6_ or C_6_-loaded micelles in 500 μL RPMI 1640 medium supplemented with 10% FBS. At predetermined time points, the cells nuclei were stained by Hoechst 33342. Then the cells were washed with cold PBS and fixed with 4% paraformaldehyde. The coverslips were mounted onto glass slides and cellular uptake was observed using confocal microscopy (Zeiss AXI0, Oberkochen, Germany). For flow cytometry assay, the cells were first seeded and incubated with different C_6_ formulations in the same way as that in the CLSM experiments. After incubation, the cells were washed with cold PBS, trypsinized and resuspended in PBS. The suspended cells were directly introduced to a flow cytometer (FACSCalibur, Becton Dickinson, Franklin Lakes, NJ, United States) equipped with a 488 nm argon ion laser. 1 × 10^4^ cells were analyzed to quantify the fluorescence intensity within the cells with blank ones as control.

### *In Vitro* Cytotoxicity and Cell Apoptosis Analysis

For cytotoxicity analysis of the as-prepared polymers, 4T1 cells were seeded in 96-well plates with a density of 1 × 10^4^ cells/well at 37°C under 5% CO_2_ and incubated for 24 h. Then the cells were treated with fresh medium containing PTX, PELA-PTX or PELA-PBAE-PTX micelles with PTX dosages from 1 to 250 nM. The cells without treatment were used as the control groups. After 48 h, the cells viability was detected by a microplate reader (Thermo MK3, Waltham, MA United States) at 570 nm using MTT assay. The viability data were analyzed with GraphPad Prism 5.01, and the IC_50_ was calculated. For cell apoptosis assay, cells were seeded in 12-well plates at 2 × 10^5^ cells/well. After 24 h, various PTX formulations at a PTX dosage of 40 nM were added to the cells for additional incubation of 24 and 48 h, respectively. Then the cells were harvested, washed twice with cold PBS, and stained with Annexin V-PE and 7-AAD (BD Biosciences, San Jose, CA, United States) for 15 min at room temperature under dark. In the end, the treated cells suspended in PBS were analyzed by flow cytometry.

### Wound Healing Assay

For evaluation of the inhibitory effect of different PTX formulations on wound healing, 4T1 cells were incubated in 12-well plates at a density of 5 × 10^5^ cells/well overnight to obtain 90% of confluence. Then two scratches (with an angle of ∼ 90° to each other) were made using a 200 μL plastic pipet tip with a ruler after removal of the medium. The cells were washed with PBS for 3 times and incubated with fresh serum free medium containing various PTX formulations with PTX dosage of 40 nM for 48 h. Images were captured on a microscope (Olympus, Japan) at 0 h and after 24 h of incubation to monitor the wound healing status. In each group, the relative percentage of wound was quantified by comparing the images of 24 h with 0 h.

### Cell Migration and Invasion Assay

For migration assay, 4T1 cells were incubated with PTX injection, PELA-PTX or PELA-PBAE-PTX at PTX dosage of 40 nM for 24 h. Then the cells were harvested and suspended in serum free medium. Afterward, the cells were seeded onto the upper Transwell chambers (Chemicon, United States) in 200 μL of serum-free medium with a density of 1 × 10^5^/mL, and 500 μL of medium containing FBS was added to the lower chambers at the same time. After 48 h of incubation, the medium on the top chambers was removed and the cells retained in the upper chambers were washed with a cotton swab. On the contrary, the cells on the surface of the lower chambers were fixed by 70% ethanol for 30 min and then stained using crystal violet for 15 min followed with PBS washing thrice. The cells were then mounted on a Leica DC 300F (Leica, Germany) microscope to evaluate the migration rate. For quantification, the cells were counted five times in random fields per chamber under the microscope. To investigate cell invasion, the matrigel was added to the upper chambers and allowed solidification overnight at 37°C. Then all the steps were similar to the above except that the cells need to degrade the matrigel layer to invade were added with 2 × 10^5^ cells to the upper chambers. The migration and invasion rate was calculated with the non-treated cells as control.

### Western Blotting Analysis

4T1 cells seeded in 6-well plates were incubated with PTX injection, PELA-PTX or PELA-PBAE-PTX at PTX dosage of 40 nM for 24 h. Then the cells were washed with cold PBS twice and incubated with lysis buffer containing 1 mmol phenylmethylsulfonyl fluoride (PMSF) for 30 min. 30.0 μg of the proteins from different samples were added to the 10% SDS-polyacrylamide gel to separate proteins with different molecular weights and then transferred to the PVDF membrane for 1 h, which was followed by blocking the membrane using 5% non-fat milk prepared with TBST solution for 1 h at room temperature and incubating with different primary antibodies of anti-uPA (Santa Cruz, CA, United States), anti-Bcl-2 (Abcam, United States), anti-twist (Abcam, United States), anti-survivin (Cell Signaling Technology, United States), anti-CD44 (Abcam, United States), anti-MMP-2 (Abcam, United States), anti-MMP-9 (Abcam, United States), and anti-actin (Sigma, United States) overnight at 4°C. Then the secondary antibodies anti-rabbit IgG, anti-goat IgG, and anti-mouse IgG (Abcam, United States) were applied to incubate with the corresponding antibodies for 45 min. After the membrane was washed with TBST for 10 min thrice, the bound antibodies were detected with enhanced chemiluminescence (ECL) reagents (Amersham, Cleveland, OH, United States) and the membrane was exposed to Hyperfilm (Amersham). The intensity of the protein were measured by Image J (National Institutes of Health) software and normalized to that of actin and expressed as relative ratios.

### Quantitative Reverse Transcriptional-Polymerase Chain Reaction (qRT-PCR)

After treatment of 4T1 cells with various PTX formulations, the total RNA was isolated using total RNA Kit (R6934, Omega Bio-tek Inc., Norcross, GA, United States) and cDNA was synthesized from 5 μg RNA in cDNA Synthesis Kit (K1622, Fermentas International Inc., Canada) according to the manufacturer’s instructions. Expression levels of uPA, Bcl-2, twist, Survivin, CD44, MMP-2, MMP-9 and actin transcript were quantified by qRT-PCR. Each PCR was performed in triplicate in a final volume of 20 μL solution. The following forward (F) and reverse (R) primers were used in this study: uPA: 5′-GCGCCTTGGTGGTGAAAAAC-3′ (F) and 5′-GACACGCATACACCTCCGTT-3′ (R); Bcl-2: 5′-GCTACCGTCGTGACTTCGC-3′ (F) and 5′-CCCCACCGAACTCAAAGAAGG-3′ (R); Twist: 5′-GGACAAGCTGAGCAAGATTCA-3′ (F) and 5′-CGGAGAAGGCGTAGCTGAG-3′ (R); Survivin: 5′-GAGGCTGGCTTCATCCACTG-3′ (F), 5′-ATGCTCCTCTATCGGGTTGTC-3′ (R); CD44: 5′-TCGATTTGAATGTAACCTGCCG-3′ (F) and 5′-CAGTCCGGGAGATACTGTAGC-3′ (R); MMP-2: 5′-ACCTGAACACTTTCTATGGCTG-3′ (F) and 5′-CTTCCGCATGGTCTCGATG-3′ (R); MMP-9: 5′-GGACCCGAAGCGGACATTG-3′ (F) and 5′-CGTCGTCGAAATGGGCATCT-3′ (R); actin: 5′-GGCTGTATTCCCCTCCATCG-3′ (F) and 5′-CCAGTTGGTAACAATGCCATGT-3′ (R). Assays were performed in triplicate with the ABI 7500 instrument (Waltham, MA, United States). All data were normalized by actin. Gene expression data was analyzed by the 2^-ΔΔCT^ method.

### Statistical Analysis

Data were processed using GraphPad Prism 5.01 software and presented as mean ± standard deviation (SD). Statistical analysis was performed using one-way analysis of variance (ANOVA). The difference was regarded statistically significant as ^∗^*P* < 0.05 and very significant as ^∗∗^*P* < 0.01.

## Results

### PTX Loaded Micelles and *in Vitro* Drug Release

PELA and PELA-PBAE were employed to incorporate PTX for evaluation of their inhibitory efficacy on the metastasis of 4T1 cells in the current study. It was demonstrated that the PTX loaded PELA and PELA-PBAE micelles were narrowly distributed with spherical shape (**Figure 1**). The diameters of PELA-PTX and PELA-PBAE-PTX micelles were 21.2 ± 0.16 and 30.8 ± 0.25 nm, respectively, which are advantageous for application as drug delivery systems with tumor treatment purposes.

**FIGURE 1:** The diameters of PTX loaded PELA-PTX micelles **(A)**, and PELA-PBAE-PTX micelles **(B)**, as determined by laser light scattering. The inset images exhibited the morphologies of the micelles captured by TEM.

The loaded PTX could be sustained released upon expose to various release medium. It should be noted that the accumulated drug release was negligible for the PELA micelles under pH 7.4 and 6.5 (**Figure 2**). However, the drug release was significantly increased from PELA-PBAE micelles under mild acidic conditions. The accumulated released drug amount during 48 h was 26.6% at pH 6.5, compared to that of 13.5% at pH 7.4.

**FIGURE 2:** *In vitro* drug release of PTX-loaded micelles in PBS at pH 7.4 and 6.5 (*n* = 3).

### *In Vitro* Cellular Uptake

Coumarin-6 (C_6_) was employed as a model probe in this study to investigate the cellular internalization of drug loaded polymeric micelles as illustrated by confocal laser scanning microscopy (CLSM) (**Figure 3**). It was demonstrated that the as-prepared polymeric cargo could help to enhance the cellular accumulation of the guest molecules, as confirmed by the stronger green fluorescence in the PELA (**Figure 3B**) and PELA-PBAE (**Figure 3C**) micellar groups, with a comparison to the weak fluorescence in the free drug group (**Figure 3A**). And stronger fluorescence was observed in PELA-PBAE group than that in PELA group.

**FIGURE 3:** Cell uptake of free C_6_ and micelles incorporated C_6_. Confocal FL images of cellular internalized C_6_ **(A)**, PELA-C_6_ **(B)**, and PELA-PBAE-C_6_ **(C)**, after 0.5 and 4 h incubation with 4T1 cells. Blue FL represents Hoechst 33342, green FL represents C_6_. **(D)** Flow cytometry analysis of mean FL intensity (*n* = 10,000 cells) in 4T1 cells incubated with C_6_, PELA-C_6_, and PELA-PBAE-C_6_ for 0.5 and 4 h, respectively. Results are presented as the mean of three measurements ± SD. ^∗^*P* < 0.05, ^∗∗^*P* < 0.01.

Moreover, the internalized content of polymer encapsulated drug increased with the elongation of incubation time, as shown in the CLSM images. The flow cytometry results also confirmed the enhanced cellular levels of endocytosed model drugs (**Figure 3D**). After 4 and 0.5 h of incubation, the internalized C_6_ in cells interior for PELA-C_6_ micelles group were 6.45 fold and 3.50 fold higher than that of free C_6_, respectively. However, for PELA-PBAE-C_6_ micelles, the accumulated C_6_ in cells were 13.78 fold and 6.77 fold higher than the free probe incubated in 4 and 0.5 h, respectively, demonstrating again of the enhanced internalization effect of the PELA-PBAE micelles.

### Cytotoxicity of PTX Loaded Micelles

At a feeding weight ratio of 0.1 of PTX to PELA and PELA-PBAE copolymers, the drug loading content of PTX was 7.5 ± 0.8% and 7.5 ± 0.7%, with corresponding loading efficiency of 82.5 ± 8.7% and 82.5 ± 8.0%, respectively, for PELA and PELA-PBAE micelles. The cellular uptake of PTX, PELA-PTX, and PELA-PBAE-PTX with elevated PTX concentration by 4T1 cells lead to the gradually increased cytotoxicity. The inhibitory effect of different PTX formulations on the cellular proliferation was conducted at pH 7.4 and 6.5, respectively. As shown in **Figure 4**, the PELA-PBAE-PTX micelles showed stronger cytotoxicity than free PTX and PELA-PTX micelles both at pH 7.4 and 6.5, which was consistent to the results in **Figure 3**, i.e., the PELA-PBAE copolymers could promote the permeation of drug loaded micelles into tumor cells cytoplasm. It should be noted that the PELA-PBAE-PTX micelles showed stronger toxicity at pH 6.5 due to the faster drug release (**Figure 2**) and the positive surface charge at acidic conditions (Data not shown). The IC_50_ values of various PTX formulations were listed in Supplementary Table 1, illustrating the enhanced inhibitory efficacy of PELA-PTX and PELA-PBAE-PTX micelles, as compared with the free drug.

**FIGURE 4:** Cytotoxicity of different PTX formulations on 4T1 cells after incubation at pH 7.4 **(A)** and 6.5 **(B)**, respectively. ^∗^*P* < 0.05.

### Cell Cycle Arrest of PTX Loaded Micelles

After being captured of the different PTX formulations by 4T1 cells, the released PTX caused cell cycle arrest in the G2-M phase (**Figure 5** and Supplementary Table 2). As shown in **Figure 5**, the G2-M population gradually increased over time, from 15% at zero time to 35% at 24 h, and to 42 and 57% for PELA-PTX and PELA-PBAE-PTX at 48 h, respectively, indicating that PTX-loaded micelles could release PTX for arrest of cell growth.

**FIGURE 5:** Cell cycle distribution of 4T1 cells. Cells were incubated in the presence of PTX **(A)**, PELA-PTX **(B)**, and PELA-PBAE-PTX **(C)**, respectively, and analyzed by flow cytometry. The equivalent PTX concentration was 40 nM.

### Wound Healing Assay and Inhibition of Cellular Metastasis

The inhibitory effect on 4T1 cells mobility by PTX formulations was analyzed by wound healing assay. It can be observed that over 73% of scratches were recovered after 48 h incubation for PTX group (**Figures 6A,D**). However, the percentages of coverage were healed 65 and 56% for PELA-PTX group and PELA-PBAE-PTX group, respectively, hinting the stronger inhibitory effect of micellar drug on tumor cells motility.

**FIGURE 6:** The inhibitory effects on motility, invasion and migration of 4T1 cells. **(A)** Wound healing images taken after treatment by PTX, PELA-PTX and PELA-PBAE-PTX with PTX dosage of 40 nM for 0 and 48 h, respectively. Representative invasion **(B)** and migration **(C)** images of cells treated with respective PTX formulations. Quantitative analysis of the inhibitory effects on cell motility **(D)**, invasion **(E)** and migration **(F)** after treatments with different PTX formulations for 24 h. Data were presented as mean ± SD (*n* = 3). ^∗^*p* < 0.05 vs. control group.

The invasion capability of 4T1 cells was analyzed by incubating the cells in an upper chamber. After incubating the cells with various PTX formulations for 24 h, the number of cells in the lower chambers was counted. As shown in **Figures 6B,E**, the inhibition rates of PELA-PTX group and PELA-PBAE-PTX group on 4T1 cells invasion were 59 and 68%, respectively, with respect to that of PTX group. Moreover, the migration rates of 4T1 cells decreased to 70 and 60% in PELA-PTX and PELA-PBAE-PTX micelles group, respectively, as compared with the PTX injection group (**Figures 6C,F**). The above results demonstrated the significant restraint ability of the micellar drugs on the invasion and migration of 4T1 cells.

### Western Blotting and qRT-PCR Analysis

After incubation with various PTX formulations, the expression of metastasis associated proteins such as uPA, twist, CD44, MMP-2 and MMP-9, and apoptosis related proteins of Bcl-2 and Survivin on 4T1 cells decreased remarkably with the strongest inhibition on the expression of the aforementioned proteins in the PELA-PBAE-PTX micelles group, respectively, as determined by Western blotting analysis (**Figure 7A**). Moreover, the mRNA levels of the respective proteins were also decreased dramatically (**Figure 7C**), demonstrating that the PTX loaded micelles were highly active in reducing the metastasis and promoting the apoptosis of 4T1 cells.

**FIGURE 7:** The effect of various PTX formulations on signaling of metastasis related proteins in 4T1 cells *in vitro*. **(A)** Western blotting analysis of the expression of uPA, Bcl-2, twist, Survivin, CD44, MMP-2 and MMP-9 on treated 4T1 cells, with actin as control. **(B)** Relative intensities of the expression of the proteins above in the cells after treatment by incubation with various PTX formulations for 24 h. **(C)** qRT-PCR determination of mRNA levels of uPA, Bcl-2, twist, Survivin, CD44, MMP-2 and MMP-9 on 4T1 cells after treatment by PTX, PELA-PTX, and PELA-PBAE-PTX micelles.

## Discussion

1-amino-4-methylpiperazine derived poly(β-amino ester) copolymer micelles were selected for incorporation of PTX to inhibit the metastasis of 4T1 cells in this study according to previous study (Chen et al., 2017). The as-prepared PELA-PBAE copolymer was demonstrated to have a sharp change in the acid-base titration curve around pH 6.4 (data not shown), which confirmed the pH sensitivity of the copolymer under tumoral microenvironments as well as cancer cells cytoplasm, which was reported to have lower pH values comparing to normal tissues (Barar and Omidi, 2013; Taylor et al., 2015). The as-prepared PTX loaded PELA and PELA-PBAE micelles were narrowly distributed with sizes around 20–30 nm (**Figure 1**). The size of the drug delivery vehicles is a crucial parameter affecting the cellular internalization as well as animal drug disposition of the drug loaded nanoparticles (Bae et al., 2005; Matsumura and Kataoka, 2009). It was demonstrated that polymer micelles with a diameter of 30 nm could efficiently penetrate through poorly permeable tumors and restrict the growth of tumors, while the increase of the micelles’ sizes could undermine their antitumor efficacy due to the difficulty in penetration through hypovascular tumors (Cabral et al., 2011).

PTX release from PELA-PBAE micelles exhibited a pH responsive profile with respect to the PELA micelles (**Figure 2**). It was reported that most solid tumors were characterized with weak acidic environments (pH 6.5∼7.4) (Taylor et al., 2015). And even lower pH values were also confirmed inside of tumor intracellular organelles (Mellman et al., 1986). Therefore, tumor microenvironment responsive drug delivery system would be highly preferred for cancer chemotherapy. Our results hinted that the PELA-PBAE micelles could be potentially used as a drug depot for pH stimulated drug release.

It was demonstrated that PELA-PBAE copolymers could improve the accumulation of more C_6_ into cellular cytoplasm, as compared with the free probe and PELA copolymers (**Figure 3**). It was reported that some polycations can intercalate into the anionic phospholipids bilayer of cellular membranes due to their protonation under mild acidic environment (Qiu et al., 2012), leading to the elevated accumulation of encapsulated drugs in cellular compartments.

The cellular uptake of PTX, PELA-PTX, and PELA-PBAE-PTX with elevated PTX concentration by 4T1 cells lead to the gradually increased cytotoxicity. It should be noted that the PELA-PBAE-PTX micelles showed stronger cytotoxicity than free PTX and PELA-PTX micelles both at pH 7.4 and 6.5 (**Figure 4**), which was consistent to the results in **Figure 3**, i.e., the PELA-PBAE copolymers could promote the permeation of drug loaded micelles into tumor cells cytoplasm. Noting that the PELA-PBAE-PTX micelles showed stronger toxicity at pH 6.5 due to the faster drug release (**Figure 2**) and the positive surface charge at acidic conditions (Data not shown). The cell cycle analysis also revealed the strongest inhibition effect was achieved by PELA-PBAE-PTX micelles, with a comparison to free PTX and PELA-PTX micelles (**Figure 5**). Moreover, the cell cycle analysis demonstrated that PTX could be released into the cytosol from polymeric micelles and was effective in reducing cell growth.

Tumor cells metastasis generally happened when cancer cells proliferated uncontrollably to produce primary heterogeneous tumors. Some circulating tumor cells from the primary cancer may invade into the circulation through lymphatic and/or blood vessels, rest at another site and form a metastatic tumor after multiplication (Menashi et al., 1998; Fayard et al., 2009). The urokinase-type plasminogen activator (uPA) contributes to the degradation of the extracellular matrix (ECM). The interaction between uPA and it specific, uPAR, was regarded as the initiator of the proteolytic cascade resulting in the degradation of basement membrane, leading to tumor invasion (Stahl and Mueller, 1994; Farina et al., 1998). Moreover, the matrix metalloproteinases (MMPs) family acts as ECM-degrading proteinases. MMP-2 and MMP-9 are two important members of MMPs involved in tumor invasion and metastasis. Meanwhile, as an epithelial-mesenchymal transition inducing transcription factor, twist has been shown to have important role in tumor metastasis, which is highly upregulated in metastatic cancer cells and various human tumors (Pai et al., 2013). On the other hand, as a member of plasma membrane glycoproteins families, CD44 has been involved in the association of cellular mitosis, migration and invasion of human carcinoma cells (Auvinen et al., 2005). In addition to the aforementioned proteins, the over expression of Bcl-2 and Survivin are prognostic markers of breast cancer, and which are closely related to the inhibition of apoptosis and promotion of cell division and angiogenesis (Jha et al., 2012; Talaiezadeh et al., 2015).

In this study, the expression of metastasis promoting proteins on 4T1 cells decreased significantly after treatment with micellar PTX, especially in the PELA-PBAE-PTX group, as shown in **Figure 7A**. The enhanced inhibitory effect of such copolymer micelles on cellular invasion and migration was most likely contributed by the downregulation of the expression of uPA, twist, CD44, MMP-2 and MMP-9 (Xu et al., 2013). Meanwhile, the corresponding anti-apoptosis proteins of Bcl-2 and Survivin were also decreased remarkably after micellar PTX treatment, implying the increased apoptosis of 4T1 cells after incubation with micellar drug. Moreover, the mRNA levels of the respective proteins were also decreased dramatically (**Figure 7C**). In accordance to the proteins levels (**Figure 7B**), the expressions of mRNA of uPA, twist, CD44, MMP-2, MMP-9, Bcl-2 and Survivin were decreased most significantly on the cells in PELA-PBAE-PTX group, suggesting again the elevated inhibition on tumor migration and invasion by the pH responsive poly(β-amino ester) copolymers.

It should be noted that the efficacy of the pH responsive polymer micelles on the inhibition of tumor metastasis on the cellular level should be verified on the animal models. Therefore, a preliminary evaluation of the inhibition of 4T1 xenograft tumor on Balb/c mice was performed in our previous research. However, the studies were not successful enough to demonstrate the enhanced therapeutic effect on tumor depression of the micellar PTX formulations, which may partially ascribed to the miss of intervention window (the tumor volumes were 100–150 mm^3^ since the treatment started in our previous evaluation), i.e., after a certain time, the therapeutic effect was not ideal even higher dosages were given (Waks et al., 2016). Nevertheless, the *in vivo* efficacy of the drug loaded pH responsive micelles needs further investigation on animal models in our future studies.

## Conclusion

In this study, pH responsive poly(β-amino ester) copolymers were prepared for inhibition of the metastatic manner of a murine breast tumor cells. The drug loaded micelles could be easily internalized with improved cytotoxicity toward 4T1 cells. The inhibitory effect of the pH responsive micelles on tumor invasion and metastasis *in vitro* were confirmed by wound healing and cell migration assay. Our findings indicate that the as-prepared polymeric micelles could be used as promising candidates for intracellular delivery of drugs for cancer chemotherapy.

## Ethics Statement

Animal studies were conducted according to the Regulation on Experimental Animals of China Academy of Chinese Medical Sciences.

## Author Contributions

JW, GD, and QY conducted the studies of preparation of PTX loaded micelles and their mechanisms for inhibition of tumor cells metastasis. HM and JC performed the characterization of control and drug loaded micelles. GZ and MD helped to measure the cytotoxicity of the as-prepared PTX formulations. HY provided assistance in experiments design and manuscript writing. QZ and YC designed the experiments and prepared the manuscript.

## Conflict of Interest Statement

The authors declare that the research was conducted in the absence of any commercial or financial relationships that could be construed as a potential conflict of interest.
